# Levels of Polycyclic Aromatic Hydrocarbons, Polychlorinated Biphenyls, and Organochlorine Pesticides in Various Tissues of White-Backed Vulture in India

**DOI:** 10.1155/2013/190353

**Published:** 2013-11-06

**Authors:** V. Dhananjayan, S. Muralidharan

**Affiliations:** ^1^Sálim Ali Centre for Ornithology and Natural History (SACON), Anaikatty, Coimbatore 641108, India; ^2^Industrial Hygiene & Toxicology Division, Regional Occupational Health Centre (Southern), ICMR Complex, Kannamangala PO, Devanahalli TK, Bangalore 562 110, India

## Abstract

This study provides information on the current status of contamination by polycyclic aromatic hydrocarbons (PAHs), polychlorinated biphenyls (PCBs), and organochlorine pesticides (OCPs) in the tissues of endangered White-backed Vulture *Gyps bengalensis* in India. Chemical analyses revealed detectable amounts of PAHs, PCBs, and OCPs. Concentration ranges of **∑**PAHs, **∑**PCBs, and **∑**OCPs in tissues were 60–2037 ng/g, 30–5790 ng/g, and 3.2–5836 ng/g wet weight, respectively. 1,1-Dichloro-2,2-bis(p-chlorophenyl)ethylene (*p,p′*-DDE) concentrations ranged from below detectable level to 599 ng/g wet weight, representing more than 90% of the total dichlorodiphenyltrichloroethane (DDT). Among the various OCPs analyzed, *p,p′*-DDE was detected most frequently. All the contaminants recorded show higher accumulation in liver than other tissues. Levels of contaminants measured in the tissues of vulture are comparable with the levels documented in a number of avian species and are lower than those reported to have caused deleterious effects. Although no threat is expected from the current level of contamination, the presence of varying levels of contaminants and their additive or synergistic toxicity is a cause of concern to vultures. Values reported in this study can serve as guideline for future research.

## 1. Introduction

Polycyclic aromatic hydrocarbons (PAHs), polychlorinated biphenyls (PCBs), and organochlorine pesticides (OCPs) are of great concern as environmental contaminants due to their persistence, lipophilicity, bioaccumulative nature [1, 2], tendency to concentrate in wildlife through food chain [2, 3], and profound consequences by way of increased reproductive dysfunction [4], increased susceptibility to diseases or other stresses, and changes in normal behavior patterns [5]. PAHs are ubiquitous environmental contaminants with high toxicity and potential carcinogenicity. As a consequence, environmental contamination by PAHs has steadily increased in recent years [6]. Although the PAHs are rapidly metabolized in birds [7], the residues of parent PAHs have been detected in bird tissues in relation to the source of combustion [8] and petroleum [4]. It has been established that an association exists between wild birds, especially birds of prey, and persistent chemical pollutants in the environment [9]. PCBs and OCPs are ubiquitous contaminants in the global environment due to their persistence and lipophilicity; they accumulate in the lipid tissues of organisms [10]. The most affected species are those which feed on contaminated food, causing population declines through long-term reproductive depression and acute poisoning [11]. Organochlorines such as hexachlorocyclohexane (HCH) and DDT still account for two-thirds of the total consumption in the country for agriculture and public health purposes, respectively [12]. Although the use of organochlorine pesticides and PCBs is restricted in India, their usage is allowed for specific purposes.

White-backed Vulture *Gyps bengalensis* was regarded as the possible commonest large raptor in the world during 1985 [13]. They feed on carcasses, often in large flocks. Indeed the number of *G. bengalensis* was considered unnaturally high because of the abundant availability of animal carcasses around human habitation in India. Prakash et al. [14] reported a decline in the population of White-backed Vulture up to 95% in its entire known distribution ranges in India during the last ten years. While Cunningham et al. [15] reported that the most likely cause of vulture decline was a novel infectious disease, Pain et al. [16] said that although there could be more than one factor responsible for such a mysterious situation, the role played by contaminants cannot be entirely ruled out. When the real reason for the vulture mortality across the country and neighbourhood continued to be elusive, Oaks et al. [17] demonstrated that the diclofenac, an anti-inflammatory drug used for treating cattle, was responsible for vulture mortality. Nevertheless, information on the residue levels of persistent contaminants, namely, PAHs, PCBs, and OCPs in vulture is necessary as they have the potential to cause mortality and population decline in birds.

Vultures, by virtue of their position at the top of the food chain, accumulate contaminants in their tissues and thus serve as sensitive indicators of environmental contamination [2]. Attention of conservationists has been on the vulnerability of birds of prey to organochlorine contaminants. Dhananjayan et al. [18] reported OCP residues in blood plasma of three species of vulture in India. It was also reported that secondary exposure to insecticide residues through feeding on contaminated carcasses is likely to be a major threat to some vulture species [19]. The objective of this study was to determine the levels of PAHs, PCBs, and OCPs in various tissues of vultures. Since there is not much information available on the residue levels of these contaminants in the tissues of vultures in India, data generated through this exercise is expected to serve as reference values.

## 2. Methods

### 2.1. Study Area and Sample Collection

Fifteen White-backed Vultures which succumbed to kite injuries in Ahmedabad (23°03.00′N to 72°58.00′E), Gujarat, were collected between January 2005 and January 2007 (Table 1). Ahmedabad is one of the cities where steel and petrochemical industries are many. Recent studies have reported prevalence of organochlorine chemical residues in blood and tissues samples of various species of birds collected in this region [18, 20–22]. Similar to the national scenario, there was a steep decline in vulture population in Gujarat between 2005 and 2007, according to surveys carried out by the Ministry of State for Environment and Forests [23]. It may be noted that people fly kites as an entertainment during a festival called *Uttarayan* which falls in January every year. While birds in thousands get injured, they die in hundreds. Samples were collected with the help of Gujarat State Forest Department and Animal Help Foundation, Ahmedabad, on opportunistic basis. Tissues or the whole carcass was air lifted to the laboratory at Coimbatore depending on the condition of the birds. Tissues, namely, brain, liver, and muscle were separated and stored in deep freezer in clean polythene vials till the time of processing.

### 2.2. Processing and Analysis of Samples for PAHs

Tissue samples (5–10 g) were digested in 6 N potassium hydroxide for 24 h at 35°C. Digestate was cooled and then neutralized with glacial acetic acid. The mixture was then extracted three times with methylene chloride, and the extracts were combined and concentrated to near dryness before reconstituting in petroleum ether for transfer to a 20 g 1% deactivated silica gel column topped with 5 g neutral alumina. PAHs were eluted using 100 mL 40% methylene chloride/60% petroleum ether followed by 50 mL methylene chloride. The eluants were concentrated using rotary flask evaporator to near dryness and redissolved in 2 mL acetonitrile. All the samples were transferred into HPLC autosampler vials for PAHs analysis as per the method followed by Hu et al. [24, 25]. All the samples were quantified for 15 components of PAHs, namely, naphthalene, acenaphthene, fluorene, phenanthrene, anthracene, fluoranthene, pyrene, benz*(a)*anthracene, chrysene, benzo[*b*]fluoranthene, benzo*(k)*fluoranthene, benzo*(a)*pyrene, dibenz*(a,h)*anthracene, benzo*(g,h,i)*perylene, and indeno(1,2,3-*cd)*pyrene using Agilent 1100 HPLC system equipped with programmable fluorescence detection at excited and emission wavelength of 260 and 500 nm, respectively. About 10 *μ*L of the sample was injected through an autosampler into C18 column (Zorbax 4.6 × 250 mm) of 5 *μ*m particle size. The temperature of the column was maintained at 20°C. Water/acetonitrile (ACN) was used as a mobile phase with a flow of 1 mL/min. The initial content of ACN was 50% and then increased into 60% (0–3 min) and 95% (3–14 min). This level was held constant for 24 min until the end of the analysis. All the results were compared with external PAHs mixture standard (AccuStandard, USA). Minimum detection limits for PAHs ranged from 3 to 10 ng/g wet weight depending on the compound. The number of spikes, duplicates, and blanks was 9% of the total number of samples analyzed. The recovery of the compounds from fortified samples (100 ng/g) ranged between 78% and 103%. Concentrations were not adjusted for per cent recovery.

### 2.3. Processing and Analysis of Samples for PCBs and OCPs

Tissues (5–10 g) were homogenized with anhydrous sodium sulphate and Soxhlet extracted with a mixture of 300 mL diethyl ether and 100 mL hexane for 7 h. After concentration through rotary evaporator, 1 mL of the aliquot was dried at 80°C to determine lipid content. The remaining extract was transferred to a 20 g Florisil-packed dry column (15 mm i.d. × 30 mm), and the solvents were dried by a gentle flow of nitrogen. Organochlorines absorbed on Florisil were eluted with a mixture of 120 mL acetonitrile and 30 mL water. The elute was transferred to a separatory funnel containing 600 mL of water and 100 mL of hexane. After partitioning, hexane layer was concentrated to 6 mL and then cleaned with equal volume of concentrated sulphuric acid. The cleaned extract was fractionated by passing through 12 g of wet Florisil column eluted with hexane (90 mL; first fraction) and then with 20% dichloromethane in hexane (150 mL; second fraction). Each faction was concentrated for analysis in gas chromatograph.

The final extracts were analyzed for 32 congeners of PCBs and the following organochlorine pesticides: isomers of hexachlorocyclohexane (HCH) (*α*-, *β*-, *δ*-, and *γ*-HCH (lindane)); DDT metabolites, namely, *p*,*p*′-DDT, 1,1-dichloro-2,2-bis(*p*-chlorophenyl)ethylene (*p*,*p*′-DDE), and *p*,*p*′-dichlorodiphenyldichloroethane (DDD); and the cyclodiene insecticides, namely, heptachlor epoxide, dieldrin, and endosulfan and its metabolites (*α*-, *β*-, and endosulfan sulfate). An aliquot (1 *μ*L) from the final extract was injected into a Hewlett Packard 5890 series II Gas Chromatograph (GC) equipped with a ^63^Ni Electron Capture Detector and a splitless injection port. The GC column employed was a DB-608 fused silica capillary column (30 m × 0.32 mm × 0.5 *μ*m thickness; J&W Scientific Inc., Folsom, CA, USA) coated with 35% phenyl methyl polysiloxane. The column oven temperature was programmed from 180°C, held for 3 min, then increased to 270°C at 10°C/min, and held for 20 min. Injector and detector temperatures were set at 250°C and 280°C, respectively. Nitrogen was used as a carrier gas with a column flow rate of 1.5 mL/min. A mixture of organochlorine pesticides (Dr. Ehrenstorfer, Germany) and a mixture of 32 PCB congeners (AccuStandard, USA) were used as standards. The concentrations of the individual compounds were quantified from the peak area of the sample to that of the corresponding external standard. Recoveries of the compounds from fortified samples (100 ng/mL) ranged from 94% to 103% and from 92% to 110% for OCPs and PCBs, respectively. Results are not corrected for per cent recovery. Analyses were run in batches of ten samples plus four quality controls (QCs) including one reagent blank, one matrix blank, one QC check sample, and one random sample in duplicate. The minimum detection limits for all the compounds analyzed were from 1 to 3 ng/g wet weight.

### 2.4. Statistical Analysis

Due to skewed distribution, organochlorine residue concentrations were log transformed to satisfy the homogeneity of variance assumption of analysis of variance (ANOVA). For the purpose of analysis, samples below the detection value were given one-half the detection limit before the comparison of the means. Means for each contaminant were compared using one-way ANOVA when at least 50% of the samples contained detectable concentrations. The probability level determining significance was *P* < 0.05 for all statistical tests. When significant differences were observed among the means, the Bonferroni multiple comparisons test was applied to determine the levels of significance. All statistical calculations were performed using statistical software SPSS student version 17.

## 3. Results

Residues of PAHs were found in all the 45 tissue samples belonging to 15 vultures. Out of 15 PAHs tested, 11 were detected in one or more tissues analyzed. Among the lower molecular weight representatives, naphthalene exhibited the highest mean concentration to *∑*PAHs (29–180 ng/g wet wt). The high molecular weight representatives were the most frequently detected, PAHs (Table 2). Phenanthrene, anthracene, chrysene, and benzo*(b)*fluoranthene were not detected in any of the tissues analyzed. The mean concentration of *∑*PAHs found in brain, liver, and muscle tissues were 363 ng/g, 812 ng/g, and 184 ng/g, wet weight, respectively. Among the tissues analyzed, liver had higher level of most of the PAHs tested, as biotransformation takes place in liver. While the total PAHs levels in brain, liver, and muscle were 176.6, 139.4, and 91.8 ng/g, respectively, during 2005, by 2007, the levels went up almost two-fold (Figure 1). However, there was no significant difference observed among the years (*P* > 0.05).

Organochlorine pesticide residues and PCB residues were detected in all the tissues of vultures (Table 3). The mean concentration of organochlorine residues in the liver tissues of White-backed Vulture was higher than that in the other tissues (*P* < 0.05). Among the various OCPs analyzed, HCH and its isomers contributed maximum to the total OCPs. The level of mean *∑*HCH among the tissues ranged from 128 to 565 ng/g. **β**-isomer of HCH accounted for the major burden of total HCH. Mean *∑*DDT among tissues ranged from 20.3 to 248 ng/g. Among the metabolites of DDT, *p,p*′*-*DDE was the most frequently detected metabolite. Its mean concentration ranged between 12.2 ng/g and 117 ng/g. The concentrations of cyclodiene insecticides were less than the other organochlorine residues. Total PCB residues in brain, liver, and muscle samples ranged from 30 to 1346 ng/g, 40 to 5790 ng/g, and 46.8 to 4063 ng/g, respectively. Similar to organochlorine pesticides, high accumulation of PCBs was found in liver tissues.

To know the temporal variation in the levels of PAHs, organochlorine pesticides, and PCBs, residue data collected between 2005 and 2007 were compared. There was no significant difference observed among the years. Hence, these concentrations could be treated as baseline values (Figure 1). Sex-wise variation was not analyzed due to small sample size.

## 4. Discussion

Analyses of results suggest that White-backed Vultures are exposed to varying levels of PAHs, and other organochlorine chemicals. It is to be noted that data on the levels of PAHs, PCBs, and pesticides in birds and with special reference to vultures in India are scarce. The absence of comparable data on residue levels in the tissues of the same species rendered direct analogies, for the majority of toxicants included in this study, extremely difficult. Therefore, this investigation was initiated to document contamination levels in vultures in India and create a database for future reference. Values cited from the literature on the levels of contaminants in tissues/serum/eggs samples of birds are not intended for direct comparisons but to provide an indication of contamination.

### 4.1. PAHs Contamination

To the best of our knowledge, this is the first report on PAHs levels in brain, liver, and muscle tissues of White-backed Vultures in India. Although PAHs are not commonly detected in the tissues of birds from noncontaminated sites, they tend to be present in very small amounts [26]. In the present study, detectable concentration of total PAHs was found in the tissues of White-backed Vulture. There are reports on the levels of PAHs in feather and plasma samples of seabirds which had fallen victims to oil spills [25] in the east coast of England. Studies on seabirds reported high concentration of PAHs accumulation through food chain [4, 27]. The source of PAHs in the tissue of birds studied in the present investigation could be through food chain accumulation. It is to be noted that Ahmedabad is one of the most industrialized cities in Gujarat, with various industries including refining operations, industrial and municipal discharges, waste oil disposal, and urban runoff. Ingestion of oil either through food or during preening is considered to be the primary source of PAHs to birds [28].

The total PAH concentration reported in the tissues in the present study are higher than the concentration reported in the whole body (120–160 ng/g) in Lesser Scaup (*Aythya affinis*),  collected from Indiana Harbor Canal, USA [4], and wild juvenile Common Eider Ducks (*Somateria mollissima*)  from the Baltic Sea [7]. Although PAH levels recorded in the present study do not reflect the extent of exposure to PAHs, the residues of parent PAH indicate that the sampling sites are contaminated with PAHs. Similar observations were reported in bird tissues from contaminated sites [4, 29]. Levels of PAHs in the present study are an order of magnitude lower than those reported in Common Guillemots *Uria aalge* which had got exposed to oil spill on the east coast of England during 2001-2002 [25].

Administration of benzo*(a)*pyrene to pigeon for 3-4 months had resulted in the formation of arterial lesions and ovarian abnormalities and eventually turned the females infertile, but apparently there were no effects on males [30]. Biomagnification of PAHs through food chain has been linked to reproductive impairment in many species of predatory birds worldwide [31]. It has been observed that the concentrations of total PAHs are considerably higher in brain than those in other tissues. Generally the contamination load in birds is related to their content and composition of prey, age, and residence time at contaminated sites [32]. Similar observations were noted in aquatic bird species, namely, Lesser Scaup, Redheads, Silver Gulls, Australian Pelicans [4, 27] and Common Guillemots [25]. Benzo*(a)*pyrene and chrysene have been shown to induce embryotoxicity in Mallards *Anas platyrhynchos*. Topical applications of eggs with benzo*(a)*pyrene (0.0336 × 10^−3^ ug/g) and chrysene (0.273 × 10^−3^ ug/g) had caused deformities and growth reductions, and in doses of 2.0 mg/kg/egg, benzo*(a)*pyrene/g and 0.273 × 10^−3^ ug of chrysene/g had caused deformities, growth reductions, and mortality [33, 34]. In doses of 2 mg/kg/egg, benzo*(a)*pyrene and indeno(1,2,3-*cd*)pyrene severely decreased survival, while chrysene caused a significant increase in lesions in embryos in Common Eider, Domestic Chicken, Turkey, and Duck [35]. Toxicity can vary with the amount and types of individual contaminants in the tissues of birds [36].

Although levels of PAHs are not likely to create lethal effect, sublethal effects such as gastrointestinal irritation, pneumonia, damage to red blood cells, immune system suppression, hormonal imbalance, impaired reproduction, and reduced growth have been reported by Albers [37] in oil ingested birds.

### 4.2. Organochlorine Pesticides

Organochlorine pesticide residues were the maximum in the liver tissues of vultures (Table 3). OCPs documented in the tissues of White-backed Vulture were lower than the levels reported in tissues of White-backed Vulture collected from the same location between 1999 and 2003 [38]. The total HCH concentrations reported in the present study are concordant with the results reported in blood plasma of three species of vulture from India [18] and lower than the levels reported in the same species collected from the urban area of Lucknow, India, during 1980 [39]. It indicates the declining trend in the environmental residue level of the compound in the Indian environment. Although the levels are not indicative of any ill effects, they are higher than the levels reported in South African Vulture [40]. Previous studies in Indian biota have also reported high levels of HCH [18, 20, 38]. There is also substantial use of *γ*-HCH in India for agricultural purpose, which is a matter of concern.

It is interesting to note that the DDE values detected in the present study are several folds lower than the values reported in the same species in Lucknow, India [39]. However, it may be noted that the levels of DDT and its metabolites detected in the present study are concordant with the results reported in tissues of the same species collected from different locations in India [38] and higher than the levels reported in the blood plasma of three species of vultures from India [18]. Although the levels of *p,p*′-DDT, *p,p*′-DDD, and *p,p*′-DDE detected in the present study were well below the levels (25 *μ*g/g of DDT) reported to be responsible for mortality of birds [41], they were higher than the levels reported in blood and tissues samples of South African White-backed Vulture [40] and serum samples of Egyptian Vulture [42]. Mean levels of total organochlorine pesticides analyzed in the present study were considerably higher than the levels reported in Cinereous Vulture (14.76 ng/g wet wt) and Eurasian Vulture (19.98 ng/g wet wt) [43]. The present study values are also far below the concentrations in eggs that were correlated with toxic effects in different species of birds (5 *μ*g/g). Higher concentration of *p,p*′-DDE in the tissues of vulture showed recent input, persistent and lipophilic nature in the environment.

The most toxic cyclodiene compound, dieldrin, was recorded in all the tissues of vulture collected from Ahmedabad. All these levels are well below the levels expected to create harmful effect to avian population [44]. However, it may be noted that the “effects range-low” (ER-L) value (i.e., the contamination level above whose adverse biological effects are occasionally observed) is listed as 0.02 *μ*g/kg for dieldrin [45]. Another cyclodiene pesticide, heptachlor epoxide, a metabolite of heptachlor, was also detected in the tissues. Residues of 0.10–0.73 *μ*g/g have been reported in Black-crowned Night-Heron [46] and 0.001 to 0.042 *μ*g/g in South African Vulture [40]. The levels recorded in the present study are higher than the LC_50_ values reported for birds [47]. The experimental study by Henny et al. [48] concluded that residues greater than 1.5 ppm were most definitely associated with decreased reproduction rates in avian species. The birds included in the study had residues of heptachlor epoxide in one or more tissues and are to be viewed with concern.

### 4.3. PCBs

The variation in contamination levels among species may be due to different feeding habitats and behaviors. The observed mean PCB concentrations were lower than those reported in birds in other countries [46]. Considerably high concentrations of total PCBs in vultures of Gujarat could be attributed to contamination due to industrial operations. Biotransformations are unlikely for the PCBs, as the majority of PCB congeners constituting the total PCB are recalcitrant in birds [49]. This pattern of high accumulation of PCB congener in avian species is contributed mainly through their food [1]. The total PCB concentration recorded in various tissues of vultures in this study is twenty fold to two hundredfold higher than the concentration reported in Black-winged Kite (29 ppb) [50], while it is two-fold higher than the levels (1600–2100 ng/g) which had shown reproductive impairment in Black Cormorant *Phalacrocorax carbo sinensis* [51] and almost similar to the levels (3600–7300 ng/g) reported to have caused tissue malformation in Double-crested Cormorant *Phalacrocorax auritus* [52].

The total PCB concentration in tissues of vultures in the present study is greater than the concentration reported in the whole body concentration of total PCB in Crested Kingfisher (160 ppb), the resident bird collected from south India, and comparable with the levels reported in a short-distance migrant, White-cheeked Tern (430–4400 ppb). It is also reported that the concentrations of PCBs in resident birds of India were less than those reported from other parts of the world. However, there has been a sign of increase in PCB concentration in resident birds, and it is assumed that PCB contamination might increase in India in the years to come due to rapid industrialization and development [50]. Additionally, unlike OCPs, PCB usage is largely related to industrial activities; therefore, higher contamination of PCBs is documented in industrial areas. Although the tissue-wise variation was not significant in the present study, liver tissues showed higher load of total PCBs. Individual PCB congeners exhibit different physicochemical properties resulting in different profile of the environmental distribution and toxicity [53].

Biotransformation may also result in lower concentrations in the liver compared with fat as the liver is an active site of biotransformation. This may occur with HCH, as reported by Moisey et al. [54], in seabirds that are known to readily biotransform both **α*-* and **γ**-HCH, but this would seem unlikely for the PCBs [49]. Hence, it may be expected that the concentration of PCBs in liver can be at higher levels. The total PCB residues in various tissues of vultures were within the range (300 to 180,000 ppb) reported in Little Egrets *Egretta garzetta* which was found dead or dying in Tokyo Bay [55]. Generally, PCBs are present at higher levels than DDE, and high concentrations of these compounds occurred in biota in water adjacent to the cities [56]. It can be suggested that the presence of petroleum-based industries in Ahmedabad might have accounted for PCB input into the environment.

## 5. Conclusion

This is the first study that documented the concentrations of PAHs, OCPs, and PCBs among various tissues of vultures in India. Among the various tissues analyzed, liver tissue recorded the maximum concentration of PAHs and other pollutants. It can be suggested that the petroleum-based industries located in Ahmedabad might have contributed to the excessive exposure of PAHs and PCBs in this species. Although the birds collected were victims to kite injuries, the concentration reported in the present study may cause sublethal effects. Although, the PCBs detected in tissues of vulture are not likely to have an impact on the demographic performance of the population as a whole, the residues may reach levels causing decreased reproduction or survival in the future, particularly when combined with other nonanthropogenic stressors such as food scarcity. In addition, the vultures normally would have more exposure to the contaminants due to their position in the food chain. Incidentally, none of the tissues are free from contaminants. Although a few experimental studies have shown the effects of PAHs on bird behavior, field assessments are invariably confounded by ecological differences between contaminated and uncontaminated sites. This study recommends continuous monitoring of persistent environmental contaminants not only in vultures but also in other species of birds.

## Figures and Tables

**Figure 1:** Variation in concentration of OCPs, PCBs, and PAHs in brain, liver, and muscle tissues of White-backed Vulture from India.

**Table 1:** Details of White-backed Vulture received from Ahmedabad, India.

S. no.	Date of collection	Location	No. of individuals	Weight (range) (kg)
1	January 2005	Ahmedabad	5 (3 M, 2 F)	5.55–6.27
2	January 2006	Ahmedabad	3 (1 M, 2 F)	3.14–4.95
3	January 2007	Ahmedabad	7 (3 M, 4 F)	4.01–6.03

**Table 2:** PAH residues (ng/g wet wt) detected in various tissues of vultures in India.

		Brain (*n* = 15)			Liver (*n* = 15)			Muscle (*n* = 15)		
PAHs		Lipid weight (%) 10			Lipid weight (%) 16			Lipid weight (%) 11		
		Mean	Range	%	Mean	Range	%	Mean	Range	%
Naphthalene	Nap	53.2	ND–246	47	180	ND–881	53	29.0	ND–123	33
Acenaphthene	Acnp	46.4	ND–212	60	ND	ND	0	ND	ND	0
Fluorene	Flu	ND	ND	0	ND	ND	0	11.8	ND–39	27
Fluoranthene	Flur	ND	ND	0	ND	ND	0	32.8	ND–144	40
Pyrene	Pyr	7.4	ND–17	47	ND	ND	0	ND	ND	0
Benz*(a)*anthracene	Bza	ND	ND	0	ND	ND	0	6.0	4.0–11	33
Benzo*(k)*fluoranthene	Bzf	15.4	ND–57	33	179	ND–876	33	ND	ND	0
Benzo*(a)*pyrene	Bzp	156	ND–645	47	307	ND–688	60	11.0	3.0–46	47
Dibenz*(a,h)*anthracene	Dbza	32.4	ND–104	27	106	ND–490	40	29.6	3.0–89	27
Benzo*(g,h,i)*perylene	Bzpe	10.6	ND–33	33	ND	ND	0	29.6	ND–219	53
Indeno(1,2,3-*cd*)pyrene	Idpy	21.6	ND–88	40	ND	ND	0	13.4	ND–47	33
Total PAHs	PAHt	363	60–941	100	812	60–2037	100	184	57–565	100

ND: not detected.

**Table 3:** Organochlorine residues (ng/g) detected in vultures in India.

Contaminants	Brain (*n* = 15)			Liver (*n* = 15)			Muscle (*n* = 15)		
	Lipid weight (%) 10			Lipid weight (%) 16			Lipid weight (%) 11		
	Mean	Range	%	Mean	Range	%	Mean	Range	%
*α*-HCH	6.9	ND–43.9	31	74.8*	ND–414	46	22.9	ND–282	38
*β*-HCH	103	ND–788	85	306	3.6–1565	100	163	3.2–1465	100
**γ**-HCH	5.7	ND–18.1	69	138*	ND–696	92	25.5	ND–168	77
**δ**-HCH	11.3	ND–43.3	15	45.6	ND–380	23	9.3	ND–76.5	38
*∑*HCH	128	1.9–893	100	565	3.6–3054	100	220	3.9–1991	100
*p,p′*-DDE	12.2	ND–68.9	77	117	4.3–599	100	86.1	ND–487	85
*p,p′*-DDD	8.2	ND–38.9	31	79.1	ND–217	46	85.5	ND–461	38
*p,p′*-DDT	3.1	ND–9.3	54	52.3	ND–263	69	12.2	ND–83.4	62
**∑**DDT	20.3	ND–117	92	248	4.3–1079	100	184	DBL–1031	85
Heptachlor epoxide	21.2	ND–93.5	38	150*	ND–1206	69	10.9	ND–29.9	54
Dieldrin	7.3	ND–43.1	23	23.2	ND–223	54	6.6	ND–45.6	46
**∑**Endosulfan	9.55	ND–56.7	15	96.1	ND–450	31	87.5	ND–384	23
**∑**OCPs	187	3.9–991	100	1083*	3.6–5836	100	509	3.2–2089	100
**∑**PCBs	359	30–1346	100	825	40–5790	100	646	46.8–4063	100

Range: (minimum–maximum), ND: below detection limit, %: percentage of sample with quantifiable level, and *: mean was significantly different from other tissues (*P* < 0.05).
